# Integrated Analysis of the Roles of RNA Binding Proteins and Their Prognostic Value in Clear Cell Renal Cell Carcinoma

This article has been retracted.

**DOI:** 10.1155/2021/5568411

**Published:** 2021-06-30

**Authors:** Bowen Wang, Haoran Zhao, Shaobin Ni, Beichen Ding

**Affiliations:** ^1^Department of Urology, The First Affiliated Hospital, Harbin Medical University, Harbin 150001, China; ^2^Department of Hepatopancreatobiliary Surgery, Harbin Medical University Cancer Hospital, Harbin, China

## Abstract

**Methods:**

We downloaded the RNA sequencing data of ccRCC from the Cancer Genome Atlas (TCGA) database and identified differently expressed RBPs in different tissues. In this study, we used bioinformatics to analyze the expression and prognostic value of RBPs; then, we performed functional analysis and constructed a protein interaction network for them. We also screened out some RBPs related to the prognosis of ccRCC. Finally, based on the identified RBPs, we constructed a prognostic model that can predict patients' risk of illness and survival time. Also, the data in the HPA database were used for verification.

**Results:**

In our experiment, we obtained 539 ccRCC samples and 72 normal controls. In the subsequent analysis, 87 upregulated RBPs and 38 downregulated RBPs were obtained. In addition, 9 genes related to the prognosis of patients were selected, namely, RPL36A, THOC6, RNASE2, NOVA2, TLR3, PPARGC1A, DARS, LARS2, and U2AF1L4. We further constructed a prognostic model based on these genes and plotted the ROC curve. This ROC curve performed well in judgement and evaluation. A nomogram that can judge the patient's life span is also made.

**Conclusion:**

In conclusion, we have identified differentially expressed RBPs in ccRCC and carried out a series of in-depth research studies, the results of which may provide ideas for the diagnosis of ccRCC and the research of new targeted drugs.

## 1. Introduction

Kidney cancer is a disease that seriously affects human health. Data show that, in 2018 alone, there were 99,200 new cases of kidney cancer in Europe; and in the past 20 years, the incidence of kidney cancer worldwide has been increasing by 2% year by year [1]. There are many types of kidney cancer, among which renal clear cell carcinoma (RCCC) is the most common type, accounting for about 80%–90% of all kidney cancer cases [2]. In recent years, with the development of medical technology, the cure rate of kidney cancer has gradually increased as well as the amount of monitoring methods. However, the diagnosis of kidney cancer mainly depends on histopathological examination, CT, and other radiographic examinations [1]. It is reported that more than half of the cases were diagnosed because of accidental examination [3]. In addition, about 30% of patients had metastatic disease during initial diagnosis [4]. Once metastatic renal cell carcinoma (MRCC) appears, the treatment will become more difficult, and meanwhile, the probability of death increases. That is why we urgently need a method that can detect kidney cancer at early stage and predict the survival time of patients. As the research on the molecular mechanism of kidney cancer continues to progress [5–8], we are now thinking about whether we can develop an effective method of early-stage diagnosis and screening based on the molecular mechanism of kidney cancer.

RNA binding proteins (RBPs) are an important class of proteins in cells and play a key role in the process of gene regulation. Except for a few RNAs that can function independently in the form of ribozymes, most RNAs perform their biological functions after combining with proteins to form RNA-protein complexes. Such RNA-protein interaction is the key to cell homeostasis. So far, more than 1500 RBP genes have been identified [9]. Further research shows that some RBPs participate in the regulation of the stability and the localization of lncRNAs [10], some ensure the accuracy of random translation by regulating mRNA [11], and some work for pre-mRNA modification [12]. There are many RBPs that can interact with the target mRNA in a sequence-and structure-dependent manner and play an important role in regulating various posttranscriptional genes such as RNA synthesis, alternative splicing, modification, transport, and translation [13]. It has been confirmed that RBP is involved in many biological processes. This also constitutes the biological basis for the occurrence and development of human diseases, which are caused by abnormal expression of RBPs.

In-depth researches on RBPs have been conducted in recent years. Some studies have shown that some RBPs, such as Pumilio, Staufen, IGF2BP, FMRP, NOVA, and ELAVL, may be related to some neuromuscular and muscular diseases [14, 15]. Others have shown that RBP to some extent works for the occurrence and development of cardiovascular diseases [16].

In the past few years, academicians have gradually found that RBP has played a role in the occurrence and development of malignant tumors [17–19], which may be related to RBP involved in a variety of posttranscriptional biological processes. However, research on cancer-related RBPs is less frequently conducted. Some results include the following: Sam68 promotes the proliferation of non-small-cell lung cancer (NSCLC) cells by activating the Wnt/*β*-catenin signaling pathway [20]; LIN28 can regulate let-7 family of miRNAs to enhance the proliferation of colon cancer cells [21]; QKI-5 accelerates tumor development by increasing the expression of miR-196b-5p [22]; and SNRPB can promote the occurrence of glioblastoma by affecting biological processes such as RNA splicing [23]. Under this circumstance, systematic studies shall be conducted for better understanding the relationship between RBP and the development of ccRCC. We downloaded RNA sequencing of renal clear cell carcinoma and patients' clinical information from the Cancer Genome Atlas (TCGA) database. Then based on bioinformatics analysis, the RBPs differentially expressed in renal cell carcinoma were found, and the biological functions involved were analyzed in detail. Also, some RBPs related to patients' prognosis were selected, based on which a model that could predict the survival time of patients was constructed. Our research has identified various RBPs associated with the prognosis of kidney cancer, some of which may become potential biomarkers of diagnosis and prognosis in the future.

## 2. Results

### 2.1. Identification of Differently Expressed RBP (DEG)

The database analysis included 539 ccRCC samples and 72 tumor-free control samples. We then conducted an in-depth study of the 1402 RBPs contained in it and finally found 125 differentially expressed RBPs, including 87 upregulated RBPs and 38 downregulated RBPs. Volcano maps (Figure 1(a)) and heat maps (Figure 1(b)) of all RBPs were constructed as well.

### 2.2. Enrichment Analysis of the Function and Pathway of Differentially Expressed RBPs

In order to further study the function of the above differentially expressed RBPs, we used *R* and related software packages for GO and KEGG pathway analysis. According to the upregulated and downregulated adjustments of RBPs, they are divided into two groups and separately analyzed. In order to show the process involved in the related RBPs more clearly, we have also made the following chart based on the analysis results. According to the GO enrichment analysis, the upregulated RBPs were significantly enriched in the following biological process (BP), namely, RNA splicing, RNA phosphodiester bond hydrolysis, nucleic acid phosphodiester bond hydrolysis, response to virus, and defense response to virus, while the downregulated RBPs were significantly enriched in regulation of RNA splicing, RNA splicing, regulation of mRNA processing, and regulation of mRNA metabolic process (Table 1).

In terms of the cellular component (CC) analysis, the upregulated RBPs were significantly enriched in spliceosomal complex, P-body, ribonucleoprotein granule, and cytoplasmic ribonucleoprotein granule, while the downregulated RBPs were notably enriched in germ plasm, pole plasm, P granule, and chromatoid body (Table 1).

The upregulated RBPs were notably enriched in molecular function (MF) process, including double-stranded RNA binding, nuclease activity, ribonuclease activity, catalytic activity, and acting on RNA, while the downregulated RBPs were significantly enriched in mRNA 3′-UTR binding, translation regulator activity, poly(U) RNA binding, and polypyrimidine tract binding (Table 1).

Besides, KEGG pathway analysis shows that upregulated RBPs mainly work in legionellosis, RNA transport, influenza A, and mRNA surveillance pathway; downregulated RBPs modulate RNA surveillance pathway, sulfur metabolism, ribosome, and 2-oxocarboxylic acid metabolism (Table 1).

### 2.3. Construction of the Protein-Protein Interaction (PPI) Network

Based on the information in the STRING database, we used Cytoscape to build a PPI network with 100 nodes and 225 edges (Figure 2(a)). In order to further identify the key modules in the coexpression network, we used the MCODE to process the coexpression network and obtained the important module as shown (Figure 2(b)). This module consists of 22 nodes and 57 edges. According to the GO enrichment analysis, the RBPs in this module involve RNA transport, protein export, RNA degradation, rRNA metabolic process, rRNA processing, mRNA catabolic process, RNA export from nucleus, ncRNA metabolic process, and translation regulator activity.

### 2.4. Screening for RBPs Related to the Prognosis of Kidney Renal Cell Carcinoma

We screened 100 important differentially expressed RBPs from the PPI network. In order to explore the relationship between these RBPs and ccRCC prognosis, we used univariate COX regression analysis to obtain 39 hub RBPs related to prognosis (Figure 3). Then for evaluating their correlation with survival time, we have screened multiple stepwise COX regression and obtained 13 hub RBPs (Figure 4). In order to determine the RBPs with the greatest potential prognosis ability among the 13 key genes, we used the ccRCC prognostic data in the LOGpc database to verify these 13 genes and finally identified 9 of the 13 RBP-encoding genes (Figure 5). These 9 RBPs can be independent predictors for ccRCC patients.

### 2.5. Construction of the Prognostic Risk Scoring Model and Survival Analysis

We used the 9 hub RBPs to construct a prognostic risk scoring model to obtain the risk score for each patient. The risk is scored by the following formula: risk score = (−0.8406 *∗* Exp TLR3) + (−0.5455 *∗* Exp PPARGC1A) + (−0.6951 *∗* Exp LARS2) + (−0.3886 *∗* Exp NOVA2) + (−0.6263 *∗* Exp RPL36A) + (−0.6496 *∗* Exp THOC6) + (0.2615 *∗* Exp RNASE2) + (0.6494 *∗* Exp U2AF1L4) + (0.5950 *∗* Exp DARS). In order to evaluate the predictive power of the model, we then divided 267 patients into low-risk group and high-risk group according to the median risk score and plotted figures after survival analysis. It is found that patients in the low-risk group have a higher survival rate than those in the high-risk group (Figure 6(a)). In addition, we made a time-dependent ROC analysis to confirm the predictive power of these 9 key RBPs (Figure 6(b)). According to the risk scoring model, the area under the curve (AUC) was 0.769, which means that it has moderate diagnostic performance. In order to confirm the evaluation ability of the model, we plotted risk score, survival status, and heat maps of expression for the above high- and low-risk groups (Figures 6(c)–6(e)). After that, to test the reliability of the above conclusions, the same method was utilized to test the other 263 patients in the TCGA database (Figure 7). The result showed that patients from the low-risk group also have a higher survival rate than those from the high-risk group. This also confirms the sensitivity and specificity of the model we built.

### 2.6. The Establishment of a Nomogram with the Nine Hub RBPs

In order to predict the survival time of ccRCC patients, we constructed a nomogram that contained all 9 RBPs signatures (Figure 8). In this nomogram, each RBP was scored between 0 and 100 according to the difference in its expression. After adding the scores of each RBP to obtain a total score, we predicted the survival rate of ccRCC patients in the first year, second year, third year, fourth year, and fifth year, which can help clinicians make better clinical decisions. Meanwhile, to look for independent prognostic factors related to ccRCC overall survival, we used COX regression analysis to perform univariate analysis and multivariate analysis on some related clinical characteristics. It is found that age, disease stage, risk score, and grade of patient all showed a significant difference with the overall survival of ccRCC patients (*P* < 0.01) (Figure 9(a)). Then, we conducted a multifactor COX regression analysis and found that patient's age, disease stage, grade, and risk score are all independent prognostic factors related to OS (*P* < 0.01). (Figure 9(b)).

### 2.7. The Expression of Hub RBPs in the HPA Database

In order to further verify the prediction accuracy of these 9 RBPs, the immunohistochemistry result of related genes was achieved in normal and tumor tissues from the Human Protein Atlas database (Figure 10). The results showed that DARS and U2AF1L4 in kidney cancer increased significantly, while the expression ability of TLR3, LARS2, NOVA2, RPL36A, and THOC6 decreased significantly. The protein expression of RNASE2 was not significantly different between tumor and normal tissue.

## 3. Discussion

Cancer is a disease that seriously affects human health and will be the leading cause of the increasing death toll as well as the most important obstacle to longer life expectancy all over the world in the 21st century [24]. Academicians have gradually deepened their research on cancer to the molecular level. In recent years, thanks to the development of microarray and high-throughput sequencing technologies, it has been found that many RBPs play a key role [25–29] in the occurrence and development of tumors, such as lung cancer [30, 31], breast cancer [32], glioma [33], and ovarian cancer [34]. However, little is known about the role of RBP in ccRCC. We hope to conduct further research to explore the biological function of RBP in ccRCC and discover its clinical significance. In this research, the ccRCC RNA sequence data were downloaded from the TCGA database, and the RBPs that were differentially expressed between tumor patients and normal people were analyzed. A functional analysis of these RBPs was performed to find out the biological process that they participated in, and a PPI network was constructed as well. Then, some RBPs related to prognosis were selected according to the clinical data and were analyzed and verified by statistical methods. We also constructed a nomogram that can predict the survival of ccRCC patients based on the selected genes. These findings may contribute to the identification of the new biomarker and provide reference to some extent to the diagnosis and prognosis of ccRCC patients.

According to the GO and KEGG pathway analysis, RBPs were enriched in the following process, including regulation of mRNA processing, regulation of mRNA metabolic process, mRNA transport, RNA splicing, RNA phosphodiester bond hydrolysis, nucleic acid phosphodiester bond hydrolysis, regulation of RNA splicing, double-stranded RNA binding, nuclease activity, ribonuclease activity, ribonuclease activity, catalytic activity, and acting on RNA. It has been proved that the posttranscriptional regulation process of genes, for instance, RNA processing and metabolism, is closely related to the occurrence and development of many diseases [35, 36]. Except for a few RNAs that can function independently as ribozymes, most RNAs combine with proteins to form RNA-protein complexes to perform their biological functions. RNA-protein interactions are associated with many diseases. In the urinary system, for example, QKI-5 enhances the stability of RASA1 mRNA, thereby inhibiting the proliferation and development of renal cancer cells [37]. In addition, RBM38 can strengthen the stability of p21 mRNA, thereby inducing cell cycle arrest in the G1 phase and controlling the development of kidney cancer [38]. HuR regulates the progress of urinary tumors by regulating mRNA transport [39]. In other cancers, reports are also common that RBP affects the occurrence and development of diseases through its participation in biological pathways. RBM3 regulates the level of SCD-circRNA 2 to influence the progress of hepatocellular carcinoma [40]. In terms of breast cancer, CRD-BP can promote the cloning of cancer cells by regulating the mRNA that acts as a code [41]; Lin28 can regulate gene expression by blocking microRNA biogenesis and thus work in the occurrence and metastasis of various cancers [42]. RBM39 in splicing regulation of its mRNA target has played a role to some extent in acute myeloid leukemia [43]. RNPC1 inhibits the metastasis of breast cancer by activating the ceRNA network related to STARD13 [44]. In addition, MSI (Musashi), IGF2BP/IMP, MEX3A, CELF1, and HUR have also been proved to play an important role in colorectal cancer [18]. A variety of RNA splicing processes exist during the translation of the human genome, and some of the RBPs presenting in spliceosome will also affect the occurrence of human diseases. For example, Sam68 can adjust the expression ratio of CyclinD1 through alternative splicing and in turn affect cancer progression [45]. In addition, KEGG analysis indicates that these RBPs may also regulate the occurrence and development of KIRC by participating in biological processes like RNA transport, mRNA surveillance pathway, sulfur metabolism, 2-oxocarboxylic acid metabolism, and ribosome pathway. Despite the great progress in the research of RBPs, given the fact that the currently discovered RBPs are less than one-tenth of all the genes that can encode proteins [9], it can be predicted that the research in this field still has great prospects in the future.

Meanwhile, we constructed a PPI network based on these differentially expressed RBPs, the key of which participated in many biological processes. And there are many reports about the role of these RBPs in cancer. As a member of Super Family 2 of helicases, DDX39B participates in almost all RNA metabolism processes, from splicing to translation as well as ribosome biogenesis [46], all of which are closely related to the occurrence and development of various human diseases [35, 36, 47]. Researches have shown that DDX39B can promote global translation and cell proliferation by upregulating the expression of precursor RNA, which may be the mechanism of DDX39B causing cancer [48]. DDX39B affects sphingolipid metabolism or N-glycan biosynthesis pathway, which results in poor prognosis of kidney cancer [49]. Also, there are detailed studies on prostate cancer [50], melanoma [51], and soft tissue sarcoma [52]. Although the correlation between most RBPs and ccRCC is still unclear, several RBPs are reported to be closely related to other cancers. As an RNA helicase, TDRD9 is involved in the biosynthesis of piRNAs and its expression is often correlated with the poor prognosis of lung adenocarcinoma. This might result from the fact that the downregulation of TDRD9 expression affects cell proliferation, causing S-phase cell cycle arrest and decreasing apoptosis [53]. TDRD 5 has the prognostic value for hepatocellular carcinoma [54]. TDRD6 is involved in chromatin body formation as well as miRNA expression and is helpful in identifying the relapse of prostate cancer [55]. RPS19 is a ribosomal protein, which can encode 40S subunit ribosomal protein. Studies have confirmed that it is significantly associated with cervical cancer and HPV infection [56]. In addition, RPS19 is significantly upregulated in prostate cancer, and it is believed to be a potential biomarker for prostate cancer [57]. There are also reports on its role in breast cancer and ovarian cancer of human beings [58]. NOP16 can regulate the size and growth of cellular by participating in rRNA synthesis and ribosome assembly. And its overexpression significantly promotes the development of breast cancer [59]. DAZL (deleted in azoospermia-like) acts as an intrinsic meiosis-promoting factor in the process of meiosis and is also an essential gene for germ cell survival [60, 61]. According to previous studies, DAZL is the key factor of germ cell tumors (GCTs) and is likely to be closely related to the occurrence of human testis cancer [62, 63]. Evidence has also shown that DAZL is related to early and preinvasive stages of cervical carcinogenesis [64].

Furthermore, we used complex statistical methods to analyze the RBPs related to the prognosis of ccRCC patients and finally obtained 9 RBPs, namely, RPL36A, THOC6, RNASE2, U2AF1L4, TLR3, PPARGC1A, DARS, LARS2, and NOVA2, most of which have been reported in detail in terms of the roles in kidney cancer and other tumors. Studies have shown that RNASE2 is a high-risk gene in ccRCC and may be related to the poor prognosis of patients [65], which is consistent with the conclusions drawn by our study. In addition, the expression level of RNASE2 is also related to the occurrence and development of prostate cancer and colorectal cancer [66, 67]. LARS2 is a leucyl-tRNA synthetase 2 located in mitochondrial, and its role in the pathogenesis has been verified, especially in cases of breast cancer [68], multiple myeloma [69], and head and neck squamous cell carcinoma [70]. In our research, LARS2 was evaluated as a low-risk gene in kidney cancer. It has been found that high expression of LARS2 may reduce the risk of lymph node metastasis in patients with nasopharyngeal carcinoma to a certain extent [71]. This conclusion is similar to our research results and may indicate that LARS2 played a similar biological role in these two cancers. As a member of the aminoacyl-tRNA synthetases (ARSs) family, DARS is defined as a high-risk gene in ccRCC. There is evidence that it is also involved in the occurrence and development of melanoma as a high-risk gene, and its high expression is significantly associated with shortened disease-free survival of melanoma patients [72]. The high expression of RPL36A is related to the pathogenesis of glioblastoma multiform [73]. In addition, RPL36A may be involved in the early development of hepatocellular carcinoma and stand as a prognostic marker for hepatocellular carcinoma [74]. It is presumed that NOVA2 worked for the metastasis of non-small-cell lung cancer (NSCLC) [75], colorectal cancer [76], and ovarian tumor [77] since its overexpression in these three cases. As an endosomal pattern-recognition receptor, TLR3 mediates innate immune response [78] and is found to induce apoptosis and thus result in oncogenesis, for instance, prostate cancer [79], non-small-cell lung cancer (NSCLC), breast cancer [80], colon cancer [81], papillary thyroid cancer [82], and nasopharyngeal carcinoma [83] as well as head and neck cancer [84]. By promoting oxidative phosphorylation and mitochondrial biogenesis, the activated PPARGC1A might accelerate metastasis [85]. Meanwhile, the high expression of PPARGC1A is closely related to the metastasis of lung cancer [86]. Alternative splicing refers to a mechanism mediated by AS factors that can cut and reconnect a gene in different ways for producing multiple mRNAs. Such mechanism can ensure proteomic and functional diversity. Studies have shown that tumor-specific isoforms produced by AS contribute to tumor development. NOVA2 as an AS factor [87] has been confirmed that it may participate in the occurrence of breast cancer by promoting epithelial-mesenchymal transition [88]. In addition, studies have shown that THOC6 is related to cancer [89, 90].

It can be seen that the prognostic RBP we screened has been mentioned and studied in terms of tumor progression, but it should also be noted that the research on these RBPs in kidney cancer is still limited. If possible, it may be valuable to further explore the potential mechanism of RBP in ccRCC. Through these studies, people may have further understanding of the pathogenesis of renal cell carcinoma or develop related targeted drugs for the treatment of the disease. Meanwhile, based on the 9 selected RBPs, we developed and validated a model that can assess the risk and survival of ccRCC patients. The statistical results also show that these genes have good diagnostic capabilities. And our nomogram may also be helpful for doctors or related personnel to clearly judge the prognostic risk of cancer patients, which may have certain value in adjusting the treatment plan of kidney cancer patients. However, our research results were not verified by *in vitro* and *in vivo* studies, which means that certain limitations may exist in our research.

In conclusion, the differentially expressed RBPs in ccRCC and the biological pathways involved were examined through bioinformatics analysis. These RBPs may be involved in the occurrence, development, or metastasis of kidney cancer. We also found out the RBPs which may be conducive to the prognosis of kidney cancer, based on which a prognostic model was constructed, the first prognostic model associated with RBPs developed for kidney cancer to our knowledge. Thus, our work is of great value for further research on the molecular mechanism of kidney cancer and the development of new targeted drugs in the future.

## 4. Materials and Methods

### 4.1. Data Acquisition and Processing

All corresponding information was downloaded from the Cancer Genome Atlas database (TCGA, https://portal.gdc.cancer.gov/). These data included RNA-seq expression dataset and relevant clinical information of 539 ccRCC samples and 72 samples of normal kidney tissue. We used a self-made Perl script to organize the clinical data. LIMMA package in *R* (http://www.bioconductor.org/packages/release/bioc/html/limma.html) was utilized to process the original data and get the expression of RBPs. Finally, we used the LIMMA package to screen for differently expressed RBPs according to the criteria that |log2 fold change (FC)| greater≥1.0 and false discovery rate (FDR) <0.05. In addition, we used the pheatmap package in *R* to construct figures of differentially expressed RBPs.

### 4.2. GO and KEGG Pathway Enrichment Analysis

We performed GO enrichment analysis and Kyoto Encyclopedia of Genes and Genomes (KEGG) pathway analysis to analyze the biological functions of differentially expressed RBPs. The GO term analysis included the biological process (BP), cellular component (CC), and molecular function (MF). In terms of GO enrichment analysis, *P* < 0.05 and FDR < 0.05 imply statistical significance; in terms of KEGG pathway analysis, *P* < 0.05 implies statistical significance.

### 4.3. PPI Network Construction

All differentially expressed RBPs were uploaded to the online STRING database (http://www.string-db.org/) for a network showing the interaction between proteins.

We used Cytoscape 3.7.1 to visualize the protein interaction network and used the included MCODE program to screen out important submodules, whose MCODE score and node number shall be more than 4, and *P* < 0.05 indicates significant difference.

### 4.4. Screening for RBPs Related to the Prognosis and Construction of the Prognostic Model

Using the survival package on *R* and presuming *P* < 0.05, we analyzed all the differentiated RBPs by the single factor of COX regression analysis for prognostic correlation analysis. Then, after conducting multiple stepwise COX regression and screening the prognostic data of KIRC related genes in the LOGpc database [90], we obtained relevant RBPs and constructed a risk model related to prognosis, in which the risk is scored by the following formula: risk score = coef1 *∗* Exp1 + coef2 *∗* Exp2 + coefx *∗* Expx. Coef is the coefficient and Exp represents the gene expression level. Finally, we evaluated the prognosis of each patient according to the risk score. In addition, according to the HR value, we divided RBPs into a low-risk group (HR less than 1) and a high-risk group (HR greater than 1) and obtained the prognosis-related RBP. Kaplan–Meier method was also used to compare the survival time of the high- and low-risk groups. We also used survival ROC on *R* for the ROC curve to better show the results we obtained.

### 4.5. Verification of Gene Expression

We use the Human Protein Atlas (HPA) database (http://www.proteinatlas.org/) to compare the expression of key RBPs.

## Figures and Tables

**Figure 1:** The differentially expressed RBPs in lung adenocarcinoma. (a) Volcano map. (b) Heat map.

**Figure 2:** Protein-protein interaction network and modules' analysis. (a) Protein-protein interaction network of differentially expressed RBPs. (b) Critical module from the PPI network. Green circles: downregulation with a fold change of more than 4; red circles: upregulation with fold change of more than 4.

**Figure 3:** Univariate COX regression analysis for the identification of hub RBPs in the training dataset.

**Figure 4:** Multivariate COX regression analysis to identify prognosis-related hub RBPs.

**Figure 5:** ccRCC prognostic data in the LOGpc database: (a) DARS, (b) LARS2, (c) NOVA2, (d) PPARGC1A, (e) RNASE2, (f) RPL36A, (g) THOC6, (h) TLR3, and (i) U2AF1L4.

**Figure 6:** Risk score analysis of the nine-gene prognostic model in the TCGA training cohort: (a) survival curve for low- and high-risk subgroups, (b) ROC curves for forecasting OS based on the risk score, (c) risk score distribution, (d) survival status, and (e) expression heat map.

**Figure 7:** Risk score analysis of the nine-gene prognostic model in the TCGA test cohort: (a) survival curve for low- and high-risk subgroups, (b) ROC curves for forecasting OS based on the risk score, (c) risk score distribution, (d) survival status, and (e) expression heat map.

**Figure 8:** Nomogram for predicting 1-, 2-, 3-, 4-, and 5-year OS of KIRC patients in the TCGA cohort.

**Figure 9:** (a) The prognostic value of different clinical parameters through single-factor COX regression analysis (*P* < 0.01). (b) The prognostic value of different clinical parameters through multiple regression analysis (*P* < 0.01).

**Figure 10:** Verification of hub RBP expression in KIRC and normal kidney tissue using the HPA database: (a) DARS, (b) TLR3, (c) LARS2, (d) NOVA2, (e) RPL36A, (f) THOC6, (g) RNASE2, and (h) U2AF1L4.

**Table 1:** KEGG pathway and GO enrichment analysis of aberrantly expressed RBPs.

	GO term	*P* value
Downregulated RBPs		
Biological processes	Regulation of mRNA metabolic process	6.07*E *−* *09
	RNA splicing	1.46*E *−* *07
	Regulation of RNA splicing	1.75*E *−* *07
	Regulation of mRNA processing	5.38*E *−* *06
	RNA splicing, via transesterification reactions with bulged adenosine as nucleophile mRNA splicing, via spliceosome	5.54*E *−* *06

Cellular component	Chromatoid body	1.58*E *−* *06
	P granule	6.24*E *−* *06
	Pole plasm	6.24*E *−* *06
	Germ plasm	6.24*E *−* *06
	Apical dendrite	0.000433273

Molecular function	mRNA 3′-UTR binding	1.07*E *−* *06
	Translation regulator activity	6.48*E *−* *06
	Poly(U) RNA binding	3.02*E *−* *05
	Polypyrimidine tract binding	4.04*E *−* *05
	Single-stranded RNA binding	0.000941036

KEGG pathway	mRNA surveillance pathway	0.006524332
	Sulfur metabolism	0.013608601
	Ribosome	0.018796706
	2-Oxocarboxylic acid metabolism citrate cycle (TCA cycle)	0.024374023
	Glyoxylate and dicarboxylate metabolism	0.040321984

Upregulated RBPs		
Biological processes	RNA splicing	3.46*E *−* *15
	Defense response to virus	5.25*E *−* *14
	RNA phosphodiester bond hydrolysis	6.81*E *−* *14
	Response to virus	3.35*E *−* *13
	Nucleic acid phosphodiester bond hydrolysis	1.68*E *−* *12

Cellular component	Cytoplasmic ribonucleoprotein granule	8.66*E *−* *11
	Ribonucleoprotein granule	1.56*E *−* *10
	P-body	6.31*E *−* *08
	Spliceosomal complex	1.30*E *−* *05
	Endolysosome membrane	2.53*E *−* *05

Molecular function	Catalytic activity, acting on RNA	1.78*E *−* *19
	Ribonuclease activity	5.30*E *−* *12
	Nuclease activity	1.20*E *−* *11
	Double-stranded RNA binding	2.17*E *−* *09
	RNA helicase activity	7.79*E *−* *08

KEGG pathway	mRNA surveillance pathway	4.13*E *−* *05
	Influenza A	7.99*E *−* *05
	RNA transport	0.000109722
	Legionellosis	0.001884052
	Spliceosome	0.003798465
	Ribosome	0.004682558
	RNA degradation	0.004769756
	RNA polymerase	0.00791322
	Toll-like receptor signaling pathway	0.010199756
	Human immunodeficiency virus 1 infection	0.012985193

## Data Availability

All corresponding information was downloaded from the Cancer Genome Atlas database (TCGA, https://portal.gdc.cancer.gov/). These data included the RNA-seq expression dataset and relevant clinical information of 539 ccRCC samples and 72 samples of normal kidney tissue. A self-made Perl script was used to organize the clinical data. LIMMA package in R (http://www.bioconductor.org/packages/release/bioc/html/limma.html) was utilized to process the original data and get the expression of RBPs. Finally, the LIMMA package was used to screen for differently expressed RBPs according to the criteria that the |log2 fold change (FC)| greater than or equal to 1≥1.0 and false discovery rate (FDR) <0.05. In addition, the pheatmap package in R was used to construct figures of differentially expressed RBPs.
